RETRACTED

# Percutaneous pedicle screw fixation combined with selective transforaminal endoscopic decompression for the treatment of thoracolumbar burst fracture

**DOI:** 10.1186/s13018-020-01946-6

**Published:** 2020-09-15

**Authors:** Zhangheng Huang, Yuexin Tong, Zhiyi Fan, Chuan Hu, Chengliang Zhao

**Affiliations:** 1 Department of Spine Surgery, Affiliated Hospital of Chengde Medical University, Chengde, 067000 Hebei China; 2 Department of Orthopedics, The Affiliated Hospital of Qingdao University, Qingdao, 266000 Shandong China

**Keywords:** Percutaneous pedicle screw fixation, Transforaminal endoscopic decompression, Thoracolumbar burst fracture, Three nerve root decompression

## Abstract

**Background:**

The objective of this study was to evaluate the feasibility, safety, efficacy, and indications of percutaneous pedicle screw fixation (PPSF) combined with selective transforaminal endoscopic decompression (TED) in the treatment of thoracolumbar burst fracture (TBLF).

**Methods:**

From August 2015 to October 2018, a total of 41 patients with single-segment TLBF (28 men and 13 women) were enrolled in this study. X-ray and computed tomography were obtained before surgery, 1 week after surgery, and 1 year after surgery to evaluate spinal recovery. In addition, we used the visual analog scale (VAS), the Oswestry Disability Index (ODI), the Japanese Orthopedic Association score (JOA), and the Frankel classification of neurological deficits to evaluate the effectiveness of the treatments.

**Results:**

The average follow-up time was 22.02 ± 8.28 months. The postoperative Cobb angle, vertebral body compression ratio, vertebral wedge angle, mid-sagittal canal diameter compression ratio, and Frankel grade were significantly improved. There were also significant improvements in the VAS (7.61 ± 1.41 vs. 1.17 ± 0.80, *P* < 0.001), ODI (89.82 ± 7.44 vs. 15.71 ± 13.50, *P* < 0.001), and JOA (6.90 ± 2.91 vs. 24.90 ± 3.03, *P* < 0.001).

**Conclusions:**

Our results showed that PPSF combined with selective TED in the treatment of TLBF had excellent efficacy, high safety, less secondary injury than other treatments, and a wide range of indications and that it could accurately distinguish patients who did not need spinal canal decompression after posterior fixation. PPSF combined with selective TED is therefore a good choice for the treatment of TLBF.

## Introduction

Thoracolumbar fractures are the most common spine fractures, with burst fractures accounting for 10–20% of these fractures [1–3]. Thoracolumbar burst fracture (TLBF) often leads to neurological dysfunction and kyphosis [4]. At present, it is generally believed that surgical treatment is preferred for burst fractures with neurological damage [5]. The main purposes of surgical treatment are to restore vertebral height, lordosis, spinal stability, and decompression of the spinal canal [6]. With the development of percutaneous pedicle screw fixation (PPSF) technology, PPSF has gained increasing recognition for thoracolumbar fractures. Its efficacy is similar to open posterior fixation, but related complications have been significantly reduced [7, 8].

RETRACTED

PPSF is mainly used for compression fractures and burst fractures without nerve damage or mild nerve damage [9]. There is still some controversy concerning the use of PPSF in the treatment of TLBF with significant neurological impairment. The controversy mainly focuses on whether it is necessary to combine it with spinal canal incision and decompression and how to choose the decompression method. Because PPSF is effective for TLBF treatment in terms of fixation and reduction, it can reset the bone mass protruding into the spinal canal, to a certain extent, and in some cases, good spinal canal recovery can be achieved without spinal canal decompression [10]. Therefore, some surgeons believe that TLBF can be treated by posterior pedicle screw fixation alone without spinal canal incision and decompression [11, 12]. Although the overall neurological functions improve significantly after surgery, there are still many cases where the neurological function is not recovered or is poorly recovered. This is because posterior pedicle screw fixation and reduction only involve indirect decompression of the spinal canal, which cannot fully decompress directly [13]. It thus may delay recovery of the damaged spinal cord and nerve function.

Based on these considerations, the current mainstream view is that TLBF with obvious neurological damage must undergo spinal canal decompression at the same time as fracture fixation and reduction. The main decompression methods are posterior decompression surgery and anterior decompression surgery [14]. Sufficient spinal canal decompression is conducive to the recovery of the damaged spinal cord and nerve function [15]. However, at the same time, spinal canal decompression involves great trauma, bleeding, and para-injury, and it may also cause secondary damage to the spinal cord and nerves. Because we cannot accurately distinguish between patients who need direct decompression and those who do not need it, all patients undergo spinal canal decompression. This indicates that this surgical method is not the perfect choice.

To solve the abovementioned complication that accurate decompression cannot be achieved, we propose the concept of PPSF combined with selective transforaminal endoscopic decompression (TED) for the treatment of TLBF. We proposed that PPSF and TED could be performed in different stages. After PPSF is performed at the first stage, the recovery of neurological function and the relief of spinal canal compression shown on postoperative computed tomography (CT) can be evaluated. For patients with satisfactory spinal canal decompression after indirect spinal canal decompression, no further spinal canal decompression is required. TED is conducted at the second stage only when patients have indications for further spinal canal decompression. This approach can achieve selective, accurate, and minimally invasive spinal canal decompression. Here, we systematically reviewed the patients treated by our method and evaluated its feasibility, safety, and effectiveness to determine the indications for the procedure and to formulate standardized treatment protocols.

RETRACTED

## Methods

### Patients

Patients who met the following inclusion criteria were included in this study: (1) A3 type in the AO classification of spinal fracture [16, 17], (2) no locked facet joint, (3) a strong will to receive surgical treatment and avoid prolonged bed rest, and (4) had follow-up at >12 months. People who met the following criteria were excluded: (1) fractures of > 2 vertebrae, (2) single-vertebra fracture with a dislocation, and (3) had follow-up at < 12 months.

### Surgery procedure

Forty-one patients underwent PPSF surgery, and fifteen of them underwent further TED surgery after PPSF. The patient was told to lie prone on a radioscopy spinal operating table with their chest, abdomen, and pelvis properly supported by gel pads. Local anesthesia plus intravenous anesthesia were performed (without tracheal intubation; the patient was conscious). After determining the skin entry point using C-arm fluoroscopy, 0.5% lidocaine was infiltrated and anesthetized to the periosteal surface, layer by layer.

The puncture needle penetrated the vertebral body through the pedicle, the position was confirmed by fluoroscopy, and a guidewire was placed. Several straight hollow pedicle screws of the appropriate size were inserted percutaneously along the guidewire. The injured vertebral body and its proximal vertebral body were implanted obliquely downward with the pedicle screws, and pedicle screws were placed in the distal vertebral bodies in a horizontal or oblique upward direction. The heads of three percutaneous screws on the same side were cohesive, and the screw tail that penetrated the injured vertebrae was slightly higher than the height of the two tails of the screws placed on the two sides of the injured vertebrae. A mild lordosis connection rod was used to fix the screws. The tail wire was tightened one by one in order to fix and reduce the injured vertebra. C-arm fluoroscopy was used to determine whether the fracture was reduced and whether the internal fixation was in the right position. The suture incision was then flushed. It was essential to review the X-rays and CT results on the first day after PPSF to evaluate the reduction and recovery of nerve function. If the nerve function was completely recovered, TED surgery was not performed. If there was still significant nerve damage or obvious hip and lower limb nerve stimulation symptoms, the patient was further treated with TED, which was performed within 5 days after the first operation.

RETRACTED

The patient lay on the contralateral side. The waist was supported by suitable lumbar padding. The skin entry point was determined by fluoroscopy. The subcutaneous tissue, fascia, and small joint capsule were injected with 0.8% lidocaine to induce local anesthesia. With the assistance of C-arm fluoroscopy, a puncture needle (size no. 16) was directly percutaneously inserted into the tip of the superior facet. Hollow manual bone drills with diameters of 4, 6, and 8 mm were used to expand the puncture and perform the foraminoplasty. We inserted a working cannula into the dilated tract through the foramen and extended the distal end of the cannula to the median part of the spinal canal until the tip of the cannula reached the posterior-superior end of the lower vertebra (Fig. 1). Decompression was performed to the intervertebral foramen, central canal, and bilateral spinal canals under the endoscope. Compressions such as fractures, fibrous rings, and ligaments in the spinal canal were removed. The “three nerve root decompression method” was used to ensure sufficient decompression on the dural sac, which meant that the entrance exiting nerve root and traversing nerve root to the inner ventral of the dural sac and contralateral traversing nerve root were fully decompressed. Endoscopic examinations ensured no compression remained, such as fractures. One drainage tube was left in place, and the surgery was completed.

**Fig. 1:** The distal end of the cannula was extended to the median part of the spinal canal (**b**), and the cannula tip reached the posterior-superior end of the lower vertebra (**a**), as visualized by C-arm fluoroscopy. The remaining fracture fragments in the spinal canal can be seen under the transforaminal endoscope (**c**, **d**)

The type of case is shown in Fig. 2.

**Fig. 2:** Imaging of the patient on admission. Lateral radiograph (**a**) shows a fracture of the L1 vertebral body. On the axial (**d**) computed tomography, the retropulsion of bone fragments into the spinal canal is evident. Magnetic resonance imaging of T2-weighted image (**b**, **c**) also showed that bone fragments had retropulsed into the spinal canal and the dural sac was severely compressed. The images of the patient were reexamined on the first day after PPSF. The sagittal (**e**) and axial (**f**) computed tomography showed that the size of the fracture fragments in the spinal canal had decreased. The images of the patient were reexamined on the 3rd day after the second operation. The sagittal (**g**) and axial (**h**) of the computed tomography showed no residual bone fragments in the spinal canal and complete decompression of the spinal cord

RETRACTED

### Assessment of clinical outcomes

We collected the data of disease histories and physical examinations of patients included in our study. A visual analog scale (VAS) was used to assess back pain of the patients preoperatively, 1 week postoperatively, and 12 months postoperatively. The Oswestry Disability Index (ODI) was used to assess disability preoperatively, 1 week postoperatively, and 12 months postoperatively. The Japanese Orthopedic Association score (JOA) was used to evaluate the clinical results preoperatively, 1 week postoperatively, and 12 months postoperatively. In addition, the Frankel classification of neurological deficits was used to assess the neurological status of the patients preoperatively and 12 months postoperatively.

### Radiographic evaluations

Radiological examinations were performed preoperatively, 1 week postoperatively, and 12 months postoperatively. The mid-sagittal canal diameter (MSD) was identified as the distance between the posterior spinal canal boundary and the anterior spinal canal boundary. The MSD compression ratio (MSDCR) was calculated according to the following formula: [(V1 + V3)/2 − V2]/(V1 + V3)/2 [18, 19]. The Cobb angle (CA), vertebral body compression ratio (VBCR), and vertebral wedge angle (VWA) were measured on the lateral X-ray (Fig. 3). The CA reflected the change of the segment curve. The VWA usually reflected the anatomical shape of the fractured vertebra.

**Fig. 3:** Measurement of radiological parameters on a lateral neutral radiograph. CA, Cobb angle; VWA, vertebral wedge angle; vertebral body compression ratio (VBCR) = [1 − (2 × body height 2)/(body height 1 + 3)] × 100

### Statistical analysis

SPSS statistical software for Windows, version 24.0 (Chicago, IL, USA) was used for statistical analysis. All data were described as the mean. Statistical *t* tests were used to compare the continuous variables pre- and postoperatively, including the VAS, ODI, JOA, Frankel grade, VWA, CA, MSDCR, and VBCR. A value of *P* < 0.05 was considered a significant difference.

RETRACTED

## Results

### Patient demographics

As shown in Table 1, a total of 41 patients (28 men and 13 women) with single-segment TLBF were included in this study from August 2015 to October 2018. Their average age was 48.93 ± 12.18 years. Surgical time was 159.24 ± 37.75 min, and in total, the average hospital stay was 10.66 ± 5.07 days and the average follow-up time was 22.02 ± 8.28 months. All patients had single-segment fractures, including one case at the T11 level, seven cases at the T12 level, 20 cases at the L1 level, nine cases at the L2 level, and four cases at the L3 level. There were 26 cases (63.4%) of type A3.1 fracture, 10 cases (24.4%) of type A3.2, and five cases (12.2%) of type A3.3.

**Table 1:** Patient demographics and perioperative parameters

Characteristic	No. of patients
Male (*n*, %)	28 (68.3)
Female (*n*, %)	13 (31.7)
Age (years)	48.93 ± 12.18
Level of fracture (*n*, %)	
T11	1 (2.4)
T12	7 (17.1)
L1	20 (48.8)
L2	9 (22.0)
L3	4 (9.8)
Type of fracture (*n*, %)	
A3.1	26 (63.4)
A3.2	10 (24.4)
A3.3	5 (12.2)
Length of stay	10.66 ± 5.07
Operation time (min)	159.24 ± 37.75
Follow-up (months)	22.02 ± 8.28

### Outcomes of the clinical data

The patient reported outcomes are shown in Table 2 and Table 3. There were significant improvements in the VAS (7.61 ± 1.41 vs. 1.17 ± 0.80, *P* < 0.001), the ODI (89.82 ± 7.44 vs. 15.71 ± 13.50, *P* < 0.001), and the JOA score (6.90 ± 2.91 vs. 24.90 ± 3.03, *P* < 0.001). According to Frankel’s classification of neurological dysfunctions, there were two cases of grade A, six cases of grade C, 19 cases of grade D, and 14 cases of grade E. All patients had no worsening of neurological function after surgery. Among the patients registered as grade D, one case was still grade D, and the rest had recovered to grade E at the 1 year follow-up. Among the patients registered as grade C, three improved to grade D and three improved to grade E. Two patients with grade A recovered to grade D at the 1 year follow-up.

**Table 2:** Functional score

	Results
VAS (back pain)	
Preoperative	7.61 ± 1.41
1 week postoperatively	3.15 ± 1.04*
12 months postoperatively	1.17 ± 0.80*
ODI (%)	
Preoperative	89.82 ± 7.44
1 week postoperatively	55.34 ± 9.31*
12 months postoperatively	15.71 ± 13.50*
JOA	
Preoperative	6.90 ± 2.91
1 week postoperatively	17.10 ± 2.54*
12 months postoperatively	24.90 ± 3.03*

*VAS* visual analog scale, *ODI* Oswestry Disability Index, *JOA* Japanese Orthopaedic Association score

*P < 0.001, there was significant difference compared with preoperative

**Table 3:** Preoperative and postoperative Frankel grades

Preoperative	12 months postoperatively				
	E	D	C	B	A
E	14				
D	18	1			
C	3	3			
B					
A		2			

RETRACTED

### Radiological data

As shown in Table 4, the preoperative CA, VWA, and VBCR were significantly reduced after surgery and remained good at 1 year of follow-up (*P* < 0.05). The 26 patients only treated with PPSF surgery had an average preoperative MSDCR value of 30.49 ± 16.25, their postoperative MSDCR decreased to 13.29 ± 8.76 (*P* < 0.001), and it remained good at the 1 year follow-up. The fifteen patients who were treated with TED surgery after PPSF had an average preoperative MSDCR of 67.39 ± 14.50. The MSDCR decreased to 4.63 ± 5.39 after two surgeries (*P* < 0.001), and remained good at the 1 year follow-up.

**Table 4:** X-radiography and CT data

	Preoperative	1 week postoperatively	12 months postoperatively
CA (°)			
A group	16.70 ± 4.62	5.59 ± 4.42***	5.57 ± 4.09^a^
B group	15.53 ± 7.59	6.49 ± 4.31***	6.78 ± 4.96^a^
VWA (°)			
A group	14.19 ± 7.89	5.96 ± 2.58*	5.67 ± 2.42^a^
B group	16.52 ± 5.74	6.77 ± 2.33***	6.95 ± 2.41^a^
VBCR (%)			
A group	39.27 ± 17.29	6.13 ± 5.25**	5.99 ± 4.98^a^
B group	37.58 ± 16.09	6.65 ± 10.84***	7.47 ± 9.06^a^
MSDCR (%)			
A group	67.39 ± 14.50	4.63 ± 5.39***	4.61 ± 5.60^a^
B group	30.49 ± 16.25	13.29 ± 8.76***	12.33 ± 7.02^a^

A group = the 15 patients who underwent TED surgery and PPSF surgery. B group = the 26 patients who underwent only PPSF surgery

*CA* Cobb angle, *VWA* vertebral wedge angle, *VBCR* vertebral body compression ratio, *MSDCR* mid-sagittal canal diameter compression ratio

*P < 0.05

**P < 0.01

***P < 0.001

^a^*P* > 0.05

## Discussion

After the occurrence of TLBF, the fractured bone mass bursts into the spinal canal and compresses the spinal cord and the ventral side of the nerve root, which is likely to cause nerve damage and further neurological dysfunction [4, 20]. Decompression surgery can help patients limit their secondary spinal cord injury and improve their neurological recovery after acute spinal cord injury [15]. At present, compared with posterior surgery, anterior surgery can achieve a more direct and complete decompression and promote better nerve recovery [14, 21]. However, the anterior approach also has some disadvantages, including the need for large surgical exposures, the risk of large vessel damage, persistent rib pain after surgery, and pulmonary complications [22]. Posterior surgery typically involves conventional posterior fixation combined with one-stage spinal canal incision and decompression. Posterior decompression is less invasive than anterior decompression but not as thorough as anterior decompression. Because of the indirect spinal decompression effect of PPSF, some TLBF can be decompressed without a spinal incision, and the symptoms of neurological deficits can be completely relieved. However, neither anterior nor posterior decompression surgery can accurately distinguish between patients who need direct decompression and those who do not need it, and unnecessary decompression is therefore performed in patients who can completely recover from their neurological deficits after posterior pedicle screw fixation. The unnecessary decompression may cause iatrogenic injury during the surgery and may increase the risk of secondary spinal cord injury.

RETRACTED

In view of these considerations, we proposed a treatment strategy that, for the first time, involved PPSF combined with selective TED. This treatment approach has the following advantages: (1) accurate and selective spinal decompression is achieved. PPSF and TED are performed at different stages, taking advantage of the indirect spinal decompression effect of PPSF. For the patients who completely recovered neurological function after PPSF, excessive decompression was avoided; for patients with poor postoperative neurological recovery, TED surgery was then performed to promote their neurological recovery. (2) Compared with both anterior surgery with direct decompression and posterior spinal canal decompression, TED surgery has the advantages of causing less injury, and its spinal canal decompression effect is similar to that of anterior decompression surgery. (3) Both PPSF and TED are minimally invasive surgeries, which have the advantages of less trauma, less bleeding, less pain, and faster postoperative recovery, and there are fewer complications related to the approach [7, 8]. (4) Local infiltration anesthesia combined with intravenous anesthesia ensured that the patient was awake during the surgery, so the patient could provide timely feedback to the surgeon to maximize the patient’s safety.

Zhao et al. [23] reported the first case of PPSF surgery combined with a transforaminal endoscope in the treatment of burst fractures. They believed that the procedure was applicable to the transverse and sagittal diameters of spinal canal bone masses not greater than 15 mm and 10 mm, respectively, and radiological evaluation of a compressed area not greater than 50% of the TLBF [23]. Based on these requirements, we further improved the TED technology and developed the three nerve root decompression method, in which the range of decompression under the percutaneous endoscope is significantly increased by decompression from the entrance exiting the nerve root and traversing the nerve root to the inner ventral of the dural sac and contralateral traversing nerve root. Here, by combining PPSF with TED, we could achieve perfect decompression and complete neurological recovery of TLBF patients with both 90% MSDCR and 90% spinal canal compression areas.

RETRACTED

Of the 41 patients with burst fractures who underwent PPSF surgery in this study, 26 of them had almost normal neurological function (14 had no nerve damage before surgery), and no further decompression of the spinal canal was required. Fifteen of these patients still had significant nerve injury or hip and lower extremity nerve irritation symptoms, so they then received TED under two-stage local infiltration anesthesia. Their lower extremity pain was completely relieved after the surgery, their neural function was also significantly restored, and there were no nerve injuries or other complications. The fifteen patients who underwent second stage TED surgery had an MSDCR of 67.39 ± 14.50 before surgery and a reduction to 4.63 ± 5.39 after surgery, indicating that their neural function was significantly restored. The spinal canal bone was quickly and completely cleared, which indicated that TED fully achieved the effect of anterior decompression with fewer injuries and complications. Our results showed that 20 of 41 cases had MSDCR < 1/3, and their symptoms were completely relieved after PPSF; 10 cases had MSDCR between 1/3 and 2/3, and 6 of them had complete relief. The other four cases required further spinal canal decompression surgery, and the 11 cases with MSDCR > 2/3 required further spinal canal decompression surgery.

We therefore believe that TLBF can be divided into three degrees according to the preoperative MSDCR: MSDCR < 1/3, degree I; 1/3 < MSDCR < 2/3, degree II; and MSDCR > 2/3, degree III. Of the fifteen patients who required secondary surgery, eleven had preoperative MSDCR > 2/3; the other four had preoperative MSDCR between 1/3 and 2/3, but the bone mass in the spinal canal was sideways and compressed more heavily than in the mid-sagittal region. Generally, for MSDCR < 1/3, no decompression is needed; for MSDCR > 2/3, decompression of the spinal canal should be performed; for 1/3 < MSDCR < 2/3, whether spinal decompression should be performed depends on the specific situation of the patient.

This finding is significant for predicting whether TLBF requires spinal canal decompression. The decision whether to perform a second stage TED surgery was mainly based on the neurological recovery of patients after PPSF. Of the fifteen patients who underwent second stage TED surgery, ten cases still had significant hip and lower limb nerve irritation symptoms and mild neurological damage after PPSF, and five cases still had significant neurological damage, and muscle strength less than grade 3 with poor function in urination and defecation. Therefore, we believe that the indications for secondary decompression surgery include (1) persistent significant neurological impairment, such as obvious muscle loss, sensory disturbances, or poor urination and defecation function; and (2) mild neurological impairment with obvious hip and lower limbs and nerve irritation symptoms remaining.

RETRACTED

In summary, PPSF combined with selective TED is suitable for all types of TLBF except dislocations. In this era of minimally invasive spine treatments, this combination treatment is expected to become the preferred method of treating TLBF. However, this study had significant limitations. First, the small sample size from a single center may have affected the conclusions. Second, this study was a retrospective study. To improve the efficacy of PPSF combined with selective TED in the treatment of TLBF and to validate the grading theory of TLBF, a larger, multicenter prospective study is needed in the future.

## Conclusion

Our results showed that PPSF combined with selective TED had excellent curative effects on TLBF with high safety, little secondary injury, and broad indications. This combination treatment accurately distinguished patients who did not need spinal canal decompression after posterior fixation. In this era of minimally invasive surgery, spine PPSF combined with selective TED may be an effective alternative to classic open surgical approaches.

## Data Availability

The datasets generated during and/or analyzed during the current study are available from the corresponding author on reasonable request.

## Abbreviations

TLBF: Thoracolumbar burst fracture
PPSF: Percutaneous pedicle screw fixation
TED: Transforaminal endoscopic decompression
CT: Computed tomography
VAS: Visual analog scale
ODI: Oswestry Disability Index
JOA: Japanese Orthopedic Association score
MSD: Mid-sagittal canal diameter
MSDCR: Mid-sagittal canal diameter compression ratio
CA: Cobb angle
VBCR: Vertebral body compression ratio
VWA: Vertebral wedge angle
